# Structural characterization of ginseng oligopeptides and anti-aging potency evaluation in *Caenorhabditis elegans*†

This article has been retracted.

**DOI:** 10.1039/d0ra06093c

**Published:** 2020-10-28

**Authors:** Qiang Luo, Jie Liu, Huailing Wang, Yi Zhou, Xiaoyu Liu, Zhigang Liu

**Affiliations:** State Key Laboratory of Respiratory Disease for Allergy at Shenzhen University, Shenzhen Key Laboratory of Allergy & Immunology, Shenzhen University School of Medicine Shenzhen 518071 China liuzhigangszu@163.com +86 755-86671911

## Abstract

The functions of ginseng polysaccharide have been widely explored, yet, the antiaging activity of ginseng oligopeptides (GOPs) has not been well explored. In the current study, seven novel GOPs were isolated, and their antiaging activity was explored in a *Caenorhabditis elegans* (*C. elegans*) model. Of interest, all the GOPs showed lifespan extending effects in *C. elegans* models. Out of the GOPs treatments, 0.75 mM GOP-1 (EHGEYE) prolonged the N2 nematodes lifespan by 42.5%. Additionally, GOP-1 had a strong free radical-scavenging activity, and up-regulated the survival of the N2 *C. elegans* under oxidative and thermal stresses. Further study revealed that GOP-1 up-regulated the transcription factor *daf-16* and *jnk-1* expressions, thus we inferred that GOP-1 promotes the lifespan and stress resistances through a JNK-1-DAF-16 pathway. The current study revealed that the ginseng oligopeptides are potential antiaging agents.

## Abstract 2

The functions of ginseng polysaccharide have been widely explored, yet, the antiaging activity of ginseng oligopeptides (GOPs) has not been well explored.

## 1. Introduction

Aging is a natural phenomenon that has common symptoms – wrinkles, dryness, darkening, pigmentation, decreased dermal thickness and a loss of elasticity. The initial theory suggested that aging, as well as the associated degenerative diseases, could be attributed to deleterious effects of free radicals on various cell components.^1^ Reactive oxygen species (ROS) are generated during cellular metabolism, primarily in the mitochondria. When the production of ROS overwhelms the antioxidant activity, damage to cellular macromolecules such as lipids, protein, and DNA may ensue.^2^ Such a state of “oxidative stress” is thought to contribute to the pathogenesis of aging. Production of free radicals is an unavoidable process in the course of cellular metabolism, and studies indicated that oxidative stress plays a fatal role in the process of aging.^3^ Studies have shown that oxidative stress and aging can be counteracted and delayed by protective antioxidant compounds: vitamins, polyphenols and amino acids.^4^ Hence, the scavenging of detrimental ROS by antioxidants may alleviate oxidative damage induced by the over-production of ROS, therefore promoting longevity and preventing aging-related disorders.^5^

The *Caenorhabditis elegans* (*C. elegans*) is widely used as an aging research model. The genome of nematodes decline behaviorally and physiologically with age in a manner has approximately 72% similarity to humans.^6^ The *C. elegans* are simple hermaphrodites with a short life-cycle (3 days for adulthood), have a large brood size (approximately 300 progeny), are relatively easy to handle, and have transparent bodies that allow one to easily observe their internal organs.^7^

As reported previously, the conserved insulin/insulin-like growth factor (IGF-1) signaling (IIS) pathway is one of the longevity-regulating pathways. The Forkhead box O (FOXO) transcription factors are key players of this pathway, which are under control of IGF-1 receptors.^8,9^ In *C. elegans*, the *daf-2* gene activation would recruit and activate the phosphoinositide 3-kinase/protein kinase B signaling cascade and results in the phosphorylation of DAF-16.^10^ Besides the IIS pathway, the Jun-N-terminal kinase-1 (JNK-1) signaling pathway is another important upstream pathway that can regulate the DAF-16 nuclear localization.

Among these co-regulators, the heat-shock-factor-1 (HSF-1) acts together with DAF-16 to activate expression of specific genes, such as genes encoding small heat shock proteins, which enhance stress resistance and longevity in the nematodes.^11^ Additionally, the p38 mitogen-activated protein kinase (PMK-1), a parallel pathway to DAF-16, also contributes to longevity of the nematodes.^12^ The FOXO family also plays a central role in regulating the stress resistance and longevity in the *C. elegans*. The best studied member of these transcription factors is DAF-16, which is one of the principal targets of the insulin-like signaling cascade, characterized by the insulin-like receptor DAF-2.^13^ In the *C. elegans*, activation of DAF-2, the nematodes homolog of IGF-1 receptor, recruits and activates the phosphoinositide 3-kinase/protein kinase B signaling cascade, which in turn results in phosphorylation of DAF-16. DAF-16 activity is further modulated by the MAPK c-Jun N-terminal kinase-1 (JNK-1). Once in the nucleus, the heat-shock-factor-1 (HSF-1) acts together with DAF-16 to activate the expression of stress-response genes, such as genes encoding small heat shock proteins, which enhance stress resistance and longevity in nematodes.^14^ Additionally, the p38 mitogen-activated protein kinase (PMK-1), a parallel pathway to DAF-16, also contributes to longevity of nematodes.^15^

As a famous traditional Chinese medicine, the ginseng is widely used in the treatments of anti-fatigue, improving the immunity and anti-cancer.^16^ Studies reported that the ginseng performed significant effect in anti-fatigue,^17^ anti-inflammation,^18^ and potent anti-allergic^19^ properties *in vivo*. Meanwhile, the ginseng polysaccharide showed strong anti-oxidative activity both *in vivo* and *in vitro*.^20^ Further, the ginseng polysaccharide also performed an interesting effects of antioxidant activities.^21^

Bioactive peptides can regulate many biological processes with relevance to aging and are widely used in anti-aging agents. For example, carnosine, also known as β-alanyl-l-histidine, is a naturally sourced dipeptide that can neutralize mixed-valence metal ions and ROS, and it is a powerful antioxidant.^22^ Palmitoyl tripeptide-5, a mimic of the thrombospondin I (TSP-I) tripeptide, can up-regulate transforming growth factor beta (TGF-β) and stimulate matrix protein production as the anti-aging agent.^23^ Acetyl hexapeptide-3 (Argireline), can inhibit the release of catecholamine (CA), noradrenaline and adrenaline by preventing the formation of the ternary SNARE complex, and it is much less toxic than botulinum toxin, making it an ideal anti-wrinkle ingredient.^24^ Although the anti-oxidant activities of ginseng polysaccharide have been extensively studied, up to now there have been no reports concerning the biological activity of ginseng oligopeptides (GOPs). Consequently, identifying the GOPs and exploring the anti-aging activity in an activity tracing and isolating method will be of great value and significance. In current study, the GOPs were isolated and amino acid sequence identified, meanwhile, the anti-aging activity and the underlying lifespan-promoting mechanism were explored in the *C. elegans* model.

## 2. Materials and methods

### 2.1 Chemicals and materials

Ginseng, the root of *Panax ginseng* C.A. Meyer (family Araliaceae) was acquired from South China Agricultural University (Guangzhou, China). The plant was authenticated the by Prof. Jie Wang, College of Pharmacy, South China Agricultural University. A voucher specimen with accession no. 2020116 was deposited in the Herbarium of the College of Pharmacy, South China Agricultural University. H_2_DCF-DA (2′,7′-dichlorodihydrofluorescein diacetate) (Sigma-Aldrich, Shanghai, China) was used as a fluorescent probe. Paraquat, was used to induce oxidative stress in nematodes (Sigma-Aldrich, Shanghai, China). All other chemicals and agents used in this study were of analytical grade and were obtained from Sigma-Aldrich (Shanghai, China) without any further purification. Bristol N2 and the transgenic strains of *mev-1* (TK22), and *daf-16* (CF1038) and *age-1* (hx546) were also obtained from the Caenorhabditis Genetics Center. Nematodes were maintained at 20 °C on plates containing Nematode Growth Medium (NGM) seeded with a live *Escherichia coli* strain OP50 as the food source according to the general procedures.

### 2.2 Isolation and identification of the GOPs

All separation procedures were performed at 4 °C. The fresh ginseng (5 kg) was minced to a homogenate mixed with the iso-propanol in a ratio of 1 : 5 (w/v) and stirred uninterrupted for 5 h. After that, the sediment was collected and freeze-dried. The defatted precipitate (212 g) was dissolved (5%, w/v) in 0.50 M phosphate buffer solution (PBS, pH 7.3). After centrifugation (10 000 × *g*, 10 min), the supernatant was collected and freeze-dried as the total protein.

The total protein (99.2 g) was fractionated using ultrafiltration with 1 kDa molecular weight (MW) cut off membranes (Millipore, China). Two peptide fractions, GOP-A (MW < 1 kDa) and GOP-B (MW > 1 kDa) were collected and freeze-dried.

#### 2.2.1 Hydrophobic chromatography

The GOP-A (47.8 g) is dissolved in 1.20 M (NH_4_)_2_SO_4_ prepared with 30 mM phosphate buffer (pH 7.3) and loaded into a phenyl sepharose CL-4B hydrophobic chromatography column (3.0 cm × 130 cm). A stepwise elution with decreasing concentrations of (NH_4_)_2_SO_4_ (1.20, 0.60 and 0 M) dissolved in 30 mM phosphate buffer (pH 7.3) in a flow rate of 2.0 mL min^−1^. Each fraction of 100 mL was collected and monitored at 280 nm. Ten fractions (GOP-A-1–GOP-A-10) were collected and the anti-aging activity in the N2 *C. elegans* was evaluated. The fraction having the most anti-aging activity was collected, and prepared for anion-exchange chromatography.

#### 2.2.2 Anion-exchange chromatography

The GOP-A-3 fraction (GOP-A-3, 4 mL, 3.42 g mL^−1^) was injected into a DEAE-52 cellulose (Sigma-Aldrich, Shanghai, China) anion-exchange column (3.0 × 130 cm) equilibrated with deionized water, and was stepwise eluted with distilled water, 0.30, 0.60, and 1.20 M (NH_4_)_2_SO_4_ solutions at a flow rate of 2.0 mL min^−1^. Each eluted fraction (100 mL) was collected and monitored at 280 nm. Eight fractions (GOP-A-3-1–GOP-A-3-8) were collected and the anti-aging activity in N2 *C. elegans* was evaluated. The fraction having the most anti-aging activity was collected, and prepared for gel filtration chromatography.

#### 2.2.3 Gel filtration chromatography

The GOP-A-3-2 fraction (GOP-A-3-2, 3 mL, 1.33 g mL^−1^) was collected and fractionated on a sephadex G-25 (Sigma-Aldrich, Shanghai, China) column (3.0 × 120 cm) in a flow rate of 2.0 mL min^−1^. Each eluate (100 mL) was collected and monitored at 280 nm, and nine fractions (GOP-A-3-2-1–GOP-A-3-2-9) were collected and the anti-aging activity in N2 *C. elegans* was evaluated. The fraction having the most anti-aging activity was collected, and prepared for Reversed Phase-High Performance Liquid Chromatography (RP-HPLC).

#### 2.2.4 RP-HPLC

The fraction GOP-A-3-2-3 (GOP-A-3-2, 1 mL, 0.42 g mL^−1^) was collected and further separated by the RP-HPLC (Agilent 1200) on a Zorbax, SB C-18 column (4.6 × 250 mm, 5 μm). The elution solvent system was composed of water–trifluoroacetic acid (solvent A; 100 : 0.1, v/v) and acetonitrile-trifluoroacetic acid (solvent B; 100 : 0.1, v/v). The peptides were separated using a gradient elution from 30% to 75% of solvent B for 50 min at a flow rate of 1.0 mL min^−1^, detection wavelength was set at 280 nm.

The separation process of the GOPs was summarized in Scheme 1.

**Scheme 1:** Isolation process of the GOPs.

In current study, seven novel GOPs were isolated and amino acid sequence identified by HPLC-ESI-MS analysis. The peptide is usually protonated under ESI-MS/MS conditions, and fragmentations mostly occur at the amide bonds because it is difficult to break the chemical bonds of the side chains at such low energy. Therefore, the b and y ions are the main fragment ions when the collision energy is <200 eV. The GOP-1 was analyzed by HPLC-ESI-MS for molecular mass determination and peptide characterization. The ion fragment *m*/*z* 763.3050 was regarded as the fragment [M + H]^+^. The ion fragment *m*/*z* 616.2372 was regarded as the y5 ion, while *m*/*z* 599.2298 was regarded as the [y5-H_2_O + H]^+^ fragment, *m*/*z* 453.1736 was regarded as the y4 ion, *m*/*z* 436.1660 was regarded as the [y4-H_2_O + H]^+^ ion and *m*/*z* 324.1306 was regarded as the y3 ion. The ion (*m*/*z* 267.1086) was the y2 ion, and ion (*m*/*z* 221.1034) was the [y2-COOH + H]^+^ fragment. On the basis of this, we concluded that the sequence of the peptide was EHGEYE (Fig. 1). Moreover, the amino acid sequences of the GOP-1 was further identified by the Edman degradation method. The rest of the GOPs were identified used the methods as the GOP-1, and the purity was detected by HPLC >98.5%. The GOPs were dissolved in DMSO (10.0 mM) and stored at 4 °C as a stock solution.

**Fig. 1:** Structure and MS/MS spectrum of GOP-1.

### 2.3 Lifespan and stress resistance

#### 2.3.1 Lifespan assay

10 gravid adult nematodes were placed on NGM plates and seeded with *E. coli* strain OP50 and laid eggs for approximate 5 h to obtain a synchronous population. Then, nematodes were removed and the plates were put back at 20 °C until the progeny reached L4 larvae. The L4 larvae nematodes were transferred to 35 mm NGM plates containing GOPs (0.10 mM) and were counted daily, and the day was counted as day 0. All experiments, except for heat shock treatment were performed at 20 °C. The nematodes that failed to move were scored as dead. Nematodes that exhibited bagging, exploded or crawled off the plates were censored. Triplicate plates were used with *N* ≥ 80 nematodes per group, and all the trails were repeated at least 3 times.

#### 2.3.2 Oxidative stress assay

Oxidative stress was assessed at 20 °C using 3 day old adult nematodes. The nematodes were incubated on treatment plates with GOP-1 0.03, 0.15 and 0.75 mM for 3 days and transferred to prepared NGM/OP50 plates, containing 1.0 mM paraquat and scored every day.

#### 2.3.3 Thermal stress assay

Thermal stress assay was performed at 35 °C using 3 day-old nematodes. The nematodes were treated on plates containing GOP-1 0.03, 0.15 and 0.75 mM for 3 days and then transferred to an incubator set to 35 °C. The number of dead nematodes was recorded every hour until approximately 50% of the controls had died.

### 2.4 Motility, brood size and intracellular ROS assays

#### 2.4.1 Motility

The L4 larvae nematodes were transferred to 35 mm NGM plates containing GOPs (0.03, 0.15 and 0.75 mM). On days 10, 13 and 16 of adulthood, nematodes were visualized. Motility classes were determined using the method reported before.^25^ A class: nematodes move spontaneously and smoothly, leaving sinusoidal and symmetric tracks; C class: nematodes only move the head or tail when prodded with a soft wire; B class: nematodes represent every behavioral class in between A and C. *N* ≥ 80 nematodes per group.

#### 2.4.2 Brood size

Nematodes were grown on NGM/OP50 plates until the late larval stage, L4, and transferred to the control plate or plates with GOP-1 (0.03, 0.15 and 0.75 mM), one nematode per plate per concentration, with *n* = 10 nematodes per group. Nematodes were then transferred every 1 day to the fresh control or GOP-1 plates until egg production had ceased. The total number of progeny was counted, and the number of progeny for each concentration was averaged.

#### 2.4.3 ROS measurement

Intracellular ROS was measured with H_2_DCF-DA as the molecular probe. The 3 day old nematodes were incubated with GOP-1 0.03, 0.15 and 0.75 mM for 3 days and then transferred to freshly prepared NGM/OP50 plates, containing 1.0 mM paraquat for 4 h. After that, all the nematodes were collected and washed with PBS for 3 times. Afterwards, the ROS level was detected.

### 2.5 Quantitative real-time PCR

The 3 day old nematodes were incubated with GOP-1 0.03, 0.15 and 0.75 mM for 3 days and then transferred to freshly prepared NGM/OP50 plates, containing 1.0 mM paraquat for 4 h. After that, the nematodes were collected and total RNA was extracted with Trizol reagent (Invitrogen), and cDNA was produced by oligo (dT) priming. The RT-PCR primers were list in Table 1. mRNA expression was performed with the method reported before.^26^ The gene expression data were analyzed using the comparative 2^−ΔΔ*C*_T_^ method, taking *actin-1* mRNA as the normalizer.

**Table 1:** The primer sequences for RT-PCR

Gene	Type	Sequence
*actin-1*	Fwd	5′-CCAGGAATTGCTGATCGTATGCAGAA-3′
	Rev	5′-TGGAGAGGGAAGCGAGGATAGA-3′
*age-1*	Fwd	5′-GAAATTAGAGCTCCACGGC-3′
	Rev	5′-TACCCTCAAGTCCACGTGTC-3′
*akt-1*	Fwd	5′-TCAAGGATGCAGCGACAATG-3′
	Rev	5′-TTGGCTGCTGATTGGTTTCC-3′
*daf-16*	Fwd	5′-CCAGACGGAAGGCTTAAAACT-3′
	Rev	5′-ATTCGCATGAAACGAGAATG-3′
*daf-2*	Fwd	5′-GGCCGATGGACGTTATTTTG-3′
	Rev	5′-TTCCACAGTGAAGAAGCCTGG-3′
*hsf-1*	Fwd	5′-TTGACGACGACAAGCTTCCAGT-3′
	Rev	5′-AAAGCTTGCACCAGAATCATCCC-3′
*jnk-1*	Fwd	5′-AGCGTGGAAGAGGATCACAA-3′
	Rev	5′-CCTCCTCCTGTTCCACTGTT-3′
*pmk-1*	Fwd	5′-GGAACTGTTTGTGCTGCTGA-3′
	Rev	5′-CGATATGTACGACGGGCATG-3′
*sod-3*	Fwd	5′-AGCATCATGCCACCTACGTGA-3′
	Rev	5′-CACCACCATTGAATTTCAGCG-3′

### 2.6 Gene deletion experiment

The N2 strain *C. elegans* were used for RNAi experiments. The plasmid for RNAi was provided by the Liu laboratory in South China University of Technology. The plasmid was transfected into *E. coli* HT115 with ampicillin (100 mg mL^−1^). *C. elegans* at the L1 stage were fed on *E. coli* HT115 containing target genes, in dishes containing isoprophylthiogalactoside (IPTG, 5 mM). *C. elegans* with a deleted *daf-16*, *jnk-1* genes were cultured and collected about 3 days after the end of the L4 larval stage. For lifespan analysis, the *C. elegans* were transferred to newly prepared dishes containing *E. coli* HT115 (*daf-16* or *jnk-1*), and the number of surviving *C. elegans* in each dish was counted every day. To determine the target genes of *daf-16* or *jnk-1*, RT-PCR analyses were conducted as described above. These experiments were repeated three times.

### 2.7 Statistical analysis

The mean lifespan and survival data were analyzed with SPSS 18 (ChicGOP, USA) Kaplan–Meier survival function and log-rank test. *N*: total number of nematodes in each individual experiment. *p* values were calculated for individual experiments, each consisting of control and experimental nematodes as the same time. All the other analyses were done using Graphpad Prism 5 (San Diego, USA). Lipofuscin accumulation was analyzed using one-way ANOVA. All values are expressed as mean ± SEM (*n* = 3). *p* < 0.05 was considered to be statistically significant.

## 3. Results

### 3.1 GOP-1 significantly prolonged the lifespan of N2 nematodes

In current study, seven novel GOPs were isolated and structure identified, further, the anti-aging activity was detected in the N2 nematodes, and the results were list in Table 2. After the 0.10 mM GOPs administration, the lifespan of the N2 nematodes were all prolonged. Interestingly, GOP-1 performed the best lifespan extending activity in N2 nematodes than the other GOPs. After the GOP-1 treatment, the lifespan was increased by 37.1% (mean lifespan: 25.5 ± 1.24 days, max lifespan: 31 days) compared to the control group (18.6 ± 1.11 days, max lifespan: 25 days). Different from the other six GOPs, we inferred that it was the glutamic acid contained in the GOP-1 performed excellent lifespan extending effect.

**Table 2:** Lifespan extending activity of GOPs^a^

Oligopeptide	Amino acid sequences	Formula	Purity (100%)	Number	Mean lifespan (days)	% of control	Maximum lifespans (days)
GOP-1	EHGEYE	C_32_H_42_N_8_O_14_	98.9	94	25.5 ± 1.24	137.1	31
GOP-2	AFEAHT	C_30_H_42_N_8_O_10_	96.2	91	23.2 ± 1.21	124.7	30
GOP-3	AHKHEW	C_37_H_50_N_12_O_9_	98.8	93	24.3 ± 1.15	130.6	29
GOP-4	LWEGHS	C_33_H_45_N_9_O_10_	99.4	95	23.4 ± 1.14	125.8	28
GOP-5	GGHTSF	C_26_H_36_N_8_O_9_	97.5	95	21.1 ± 1.21	113.4	27
GOP-6	YGHEKF	C_37_H_49_N_9_O_10_	98.2	91	22.5 ± 1.20	120.9	27
GOP-7	SLAHRF	C_33_H_51_N_11_O_8_	98.1	94	21.3 ± 1.22	114.3	27
GSH	GSH	C_10_H_17_N_3_O_6_S	96.4	92	23.6 ± 1.24	126.8	29
Control	—	—	—	93	18.6 ± 1.11	100.0	25

a All values are expressed as mean ± SEM (*n* = 3). The GSH was used as the positive control agent.

The *Escherichia coli* growth may affect the diet of the nematodes, and then affect the lifespan. However, we observed that all the GOPs did not infect the growth cycle of the *Escherichia coli* strain OP50 under 8.0 mM (data were not listed in current study). So, the possibility that the *Escherichia coli* growth affected the lifespan of the nematodes was ruled out.

The wild-type N2 nematodes have a mean lifespan of 14–28 days at 20 °C. Under our standard laboratory conditions, wild-type N2 nematodes lived an average of 18.6 ± 1.11 days (maximum of 25 days). After treated with GOP-1 (0.03, 0.15 and 0.75 mM), starting at the L4 larvae stage, the mean lifespans of nematodes were increased to 19.9 ± 1.54 days (maximum of 26 days), 25.7 ± 1.76 days (maximum of 31 days) and 26.5 ± 1.83 days (maximum of 32 days), increased by 6.99%, 38.2% (*p* < 0.05) and 42.5% (*p* < 0.05), respectively, in a statistically significant, dose-dependent manner (Fig. 2 and Table 3).

**Fig. 2:** GOP-1 extends the lifespan of N2 nematodes. L4 N2 nematodes (*N* ≥ 80 each group) were treated 0.03, 0.15 and 0.75 mM GOP-1 for 3 days. After that the nematodes were transferred to the NGM plates and the survival was monitored as experimental design. The experiment was repeated at least 3 times.

**Table 3:** Effect of GOP-1 on the lifespan of N2 nematodes^a^

Groups	Number	Mean lifespan (days)	% of control	Maximum lifespans (days)
Control	85	18.6 ± 1.11	100.0	25
GOP-1 0.03 mM	83	19.9 ± 1.54	106.9	26
GOP-1 0.15 mM	85	25.7 ± 1.76	138.2	31
GOP-1 0.75 mM	84	26.5 ± 1.83	142.5	32

a All values are expressed as mean ± SD (*n* = 3).

### 3.2 GOP-1 enhanced motility and reduced the intracellular ROS levels

The ROS are intermediates formed during electron reduction of molecular oxygen. The free radical theory of aging hypothesized that ROS are implicated as being important in the pathogenesis in a wide range of diseases or pathological processes, including various forms of cancer, type 2 diabetes mellitus,^27^ atherosclerosis and aging.^28^ There are many factors to which the organism is exposed like smoke, microorganisms, or UV radiation, leading to the generation of ROS. Some agents such as paraquat, UV-radiation and lipopolysaccharide (LPS) are usually used to induce oxidative damage and premature aging.^29^ The antioxidants constitute a major cell defense against acute oxygen toxicity and protect membrane components against damage caused by the ROS. In current study, to explore how GOP-1 improved the stress resistance ability of the nematodes under environmental stress, the ROS scavenging activity of GOP-1 was evaluated, and the results were list in Fig. 3A.

**Fig. 3:** GOP-1 down-regulated the intracellular ROS production in N2 nematodes. (A) N2 nematodes showed different intracellular ROS levels in response to 1.0 mM paraquat when treated with the GOP-1. The ROS level in the control group was set as 1. Significant differences from the control group were observed in the GOP-1 treated groups (##*p* < 0.01, *vs.* control, *p < 0.05, **p < 0.01, *vs.* paraquat). (B) There were no significant differences in the number of total progeny between the GOP-1-treated groups and control group. (*N* = 10 nematodes per group).

Compared to the control group, the ROS level was increased by 539% after the paraquat treatment (*p* < 0.01). Interestingly, after the 0.03, 0.15 and 0.75 mM GOP-1 treatments, the ROS levels were reduced by 23.4%, 39.9% (*p* < 0.05) and 70.7% (*p* < 0.01), respectively. We inferred that GOP-1 is a significant ROS scavenger *in vivo*.

An increase in lifespan is often correlated with a decrease in the reproductive capacity. To test whether the GOP-1 decreases the reproductive capacity of the N2 nematodes, we detected the brood sizes of N2 nematodes under GOP-1 treatments. As shown in Fig. 3B, there were no significant differences between GOP-1 treated groups and the control group.

Studies reported that the increase in lifespan is usually accompanied by an overall improvement in health and vitality. Here, we explored whether the increase in lifespan of N2 nematodes is accompanied by the vitality when treated with the GOP-1. The decline in motility on day 10 was delayed significantly in nematodes treated with the GOP-1 (Fig. 4). On day 10, most nematodes in the GOP-1 groups continued to move spontaneously, but there was a gentle difference in (class A) motility among the control and GOP-1 0.20 mM (*p* < 0.05), 1.00 mM (*p* < 0.05) treatment groups (Fig. 4). By day 13, nematodes treated with GOP-1 0.20 mM had significantly (*p* < 0.05) more high-motility (class A and B) individuals (76.3%) than the control group (55.2%).

**Fig. 4:** Effect of GOP-1 on motility of (A) day 10, (B) day 13 and (C) day 16 in N2 nematodes. Motility was classified into three classes: (A): nematodes moved spontaneously; (B): nematodes required prodding to stimulate movement; (C): nematodes only moved their heads in response to a gentle touch. The decline in motility on day 16 was significantly delayed in nematodes treated with GOP-1 0.75 mM. (*N* ≥ 40 nematodes per group for day 10 and 13; *N* ≥ 15 for day 16).

By day 16, the dose-dependent effects on motility were clearly evident (Fig. 3), such that 70.6% of the control group would barely move (class C), while 38.8% of the GOP-1 1.0 mM treatment group still moved spontaneously (class A).

### 3.3 GOP-1 enhanced the stress resistance of nematodes

Studies demonstrated that increased lifespan often correlates with increased anti-oxidant stress resistance.^30^ Paraquat has been widely used to induce oxidative damages in nematodes for stress study. In current study, the lifespan of the N2 nematodes in the paraquat group was 5.69 ± 0.42 days (maximum of 8 days); compared to the control group (18.6 ± 1.11 days, max lifespan: 25 days), the lifespan was decreased by 69.4% (Fig. 5). The results indicated that the nematodes were suffered a fatal damage induced by the paraquat. Of interest, the GOP-1 increased the lifespan of the nematodes. Compared to the paraquat group, the nematodes in the 0.03, 0.15 and 0.75 mM GOP-1 treatment groups were 6.87 (maximum of 8 days), 7.94 (maximum of 10 days), and 9.53 days (maximum of 12 days), respectively. These represented statistically significant increases in the lifespan of 20.7%, 39.5% (*p* < 0.05) and 67.5% (*p* < 0.05) over the paraquat group (Fig. 5). However, the lifespan of TK22 and CF1038 nematodes under the GOP-1 treatments showed no significant difference.

**Fig. 5:** Effect of GOP-1 on resistance to oxidative stress. Nematodes were treated with GOP-1 0.03, 0.15 and 0.75 mM for 3 days at 20 °C, then, exposed to the paraquat as the experimental design (*N* ≥ 80 nematodes, ##*p* < 0.01, *vs.* control, *p < 0.05, **p < 0.01, *vs.* paraquat, log-rank test).

Nematodes were placed in a 35 °C thermal shock chamber and monitored until approximately 50% of the N2 nematodes had died (11.3 h). Of interest, 55.7%, 60.6% and 65.4% of the nematodes in GOP-1 0.03, 0.15 and 0.75 mM treated groups were still alive at that time. Nematodes that have a mutation in *age-1*, the PI3 kinase, are more resistant to heat stress, were used as a negative control and survived at a 79.3% rate; *daf-16* nematodes, which are more sensitive to heat stress, were used as a positive control and had a 40.6% survival rate (*p* < 0.05; Fig. 6). Apparently, GOP-1 could enhance the stress-resistance ability of nematodes under thermal and oxidative stresses.

**Fig. 6:** Effect of GOP-1 on resistance to thermal stress in nematodes. Nematodes were treated with 0 (control), GOP-1 0.03, 0.15 and 0.75 mM for 3 days at 20 °C and exposed to thermal stress on the fourth day. (*N* ≥ 100 nematodes, *p < 0.05, two-sample *t*-test). Each experiment is representative of three independent trials.

### 3.4 GOP-1 regulated the stress resistance associated gene expressions

To explore the possible mechanism of GOP-1 extending the nematodes lifespan, we detected the effects on the mutant nematodes, which are short-lived due to the oxidative stress. We then focused on the insulin/insulin-like growth factor-1 (IGF1) signaling pathway, in which the translocation of the FOXO transcription factor DAF-16 into the nucleus is believed to modulate stress response and longevity of the nematodes. Due to the important role of DAF-16 in this pathway, we assessed the effects of the GOP-1 on the life span of a mutant CF1038 strain, which lacks of daf-16.

As a result, GOP-1 failed to extend the life span of TK22 and CF1038 nematodes, indicating that endogenous signaling pathways rather than the antioxidative activity alone are required to promote lifespan (Fig. 5). Taken together with the results on the N2 and TK22 nematodes, our data clearly suggest that signaling pathways are definitely required to promote longevity, and DAF-16 is indispensable for the life span-extending effects of the GOP-1.

To investigate the possible underlying mechanisms of GOP-1 extending nematodes lifespan, we performed quantitative real-time PCR experiments to assess the expressions of *daf-2*, *age-1*, *akt-1*, *daf-16*, *sod-3*, *jnk-1*, *hsf-1* and *pmk-1*. As seen in Fig. 7, GOP-1 up-regulated the expressions of *daf-16*, whereas the expression of *age-1*, *akt-1*, *daf-2* and *sod-3* remained unchanged. The result indicated that the GOP-1 promoted the longevity of *C. elegans via* modulation of DAF-16. Intriguingly, it was observed that GOP-1 up-regulated the expression of *jnk-1*. In addition, GOP-1 also up-regulate the expression of *hsf-1* which cooperates with DAF-16 in regulating stress-response genes. Further, we found that the expression of *pmk-1* was not changed after GOP-1 treatment. Collectively, our results suggest that the GOP-1 may promote the *C. elegans* lifespan and stress resistance through a JNK-1-DAF16 pathway. This result suggested that the GOP-1 are apparently taken up and exhibit *in vivo* antioxidant activities to reduce the burden of oxidative stress.

**Fig. 7:** Gene expressions of N2 nematodes under GOP-1 treatment. The mRNA levels of corresponding genes were determined by the quantitative RT-PCR in *C. elegans* with GOP-1 treatments. RT-PCR was performed using 2^−ΔΔ*C*_T_^ method and normalized to the expression of gene *actin-1*. In each experiment, control and experimental *C. elegans* were conducted in parallel and repeated in three independent trials. Bars represent the mean value of three independent experiments (*p < 0.05, **p < 0.01, *vs.* control).

### 3.5 GOP-1 could not increase lifespan of *C. elegans* RNAi (*daf-16* or *jnk-1*)

The *daf-16* and *jnk-1* gene regulates stress resistance and lifespan through the insulin signalling pathway (IIS). To determine whether GOP-1 could affect the lifespan of *C. elegans* deficient in *daf-16* and *jnk-1*, we treated RNAi (*daf-16* or *jnk-1*) *C. elegans* with GOP-1 for 5 days from the start of the young adult stage and examined their lifespan (Table 4). The RNAi method effectively silenced *daf-16* or *jnk-1*. Under our normal standard laboratory conditions, RNAi (*daf-16*) *C. elegans* lived an average of 15.2 ± 0.51 days, and RNAi (*jnk-1*) *C. elegans* lived an average of 14.4 ± 0.43 days. After treatment with GOP-1, the mean lifespan of these mutants (*daf-16* or *jnk-1*) did not significantly increase.

**Table 4:** Effect of GOP-1 on the lifespan of *C. elegans* in RNAi (*daf-16* or *jnk-1*)^a^

Groups	Number	Mean lifespan (days)	% of control	Maximum lifespans (days)
**Control (*daf-16*)**	98	15.2 ± 0.51	100.0	18
GOP-1 0.03 mM (*daf-16*)	87	14.9 ± 0.51	98.2	17
GOP-1 0.15 mM (*daf-16*)	85	14.7 ± 0.49	96.7	17
GOP-1 0.75 mM (*daf-16*)	79	14.5 ± 0.48	95.4	16
**Control (*jnk-1*)**	99	14.4 ± 0.43	100.0	17
GOP-1 0.03 mM (*jnk-1*)	81	14.3 ± 0.39	99.3	16
GOP-1 0.15 mM (*jnk-1*)	85	14.1 ± 0.41	97.9	16
GOP-1 0.75 mM (*jnk-1*)	86	14.0 ± 0.41	97.2	15

a All values are expressed as mean ± SD (*n* = 3). From the beginning of synchronization, it is recorded as day 1.

## 4. Discussion

Natural products represent an extraordinary source of novel chemical entities for potential anti-aging agents. Further, the natural products performed excellent activities in delaying age-related decline and extending lifespan of the nematodes.^31^ Here, we reported that the antioxidant peptide isolated from ginseng possess promising anti-aging activities observed in *C. elegans*, a widely used model animal in aging research. To our knowledge, this is the first report describing the antiaging effects of GOPs in *C. elegans*, adding a novel source to the antiaging natural products. We found that the GOPs can significantly increase the lifespan of the wild type N2 nematodes under normal culture conditions. Particularly, GOP-1 exhibited the strongest longevity-promoting effect. At the concentration of 0.75 mM, GOP-1 significantly extended the mean lifespan of *C. elegans* by 42.5%.

Numerous studies have shown that longevity-promoting activity of natural product is correlated to their antioxidant activities. Interestingly, the GOP-1 show potent *in vivo* antioxidant potentials in *C. elegans*. We found that the GOP-1 significantly decreased endogenous ROS levels in the N2 nematodes (Fig. 3A), indicating that the GOP-1 is indeed *in vivo* antioxidants in *C. elegans*. More intriguingly, the GOP-1 markedly increased the lifespan of *C. elegans* under oxidative stress induced by the strong pro-oxidant paraquat (Fig. 4A), suggested that GOP-1 can protect the *C. elegans* from severe oxidative stress.

Hormesis mechanisms have been found in lifespan extension and stress resistance of *C. elegans* upon treatments with antioxidants. As such, we speculate that the protective effect of the GOP-1 in *C. elegans* under oxidative stress is likely due to stress hormesis, in which endogenous antioxidant response pathways are activated by antioxidants. However, we observed that GOP-1 failed to extend the mean life span of TK22 and CF1038 mutant *C. elegans* (Fig. 5), which are short-lived due to a high endogenous oxidative flux. This finding highly suggested that endogenous signaling pathways other than only direct antioxidant mechanism are involved in the life span extension of *C. elegans* induced by the GOP-1.

To further explore the antiaging potential mechanism of the GOP-1, we focused on the IIS pathway, which is a pivotal longevity-regulating pathway conserved in both *C. elegans* and mammals. In *C. elegans* the major longevity promoting transcription factor DAF-16 is a central player in the IIS pathway. In contrast to the effect observed in N2 *C. elegans*, GOP-1 failed to extend the life span of the mutant strain lacking DAF-16, implying that the GOP-1 extend life span of *C. elegans* through a mechanism that is mediated by DAF-16. The nuclear translocation of DAF-16 is a key step in the IIS pathway, as it regulates the transcription of a number of longevity- and stress tolerance-associated genes. However, we did not observe alterations of expression of *daf-2*, *age-1* and *akt-1* which are key upstream elements of IIS pathway in the *C. elegans* treated by the GOP-1. It suggested that IIS pathway may not contribute to the longevity promotion effect of GOP-1. In addition, by using quantitative RT-PCR we found that the transcriptional level of the *daf-16* in N2 *C. elegans* can be markedly up-regulated by GOP-1 about 3.92-fold, suggesting that DAF-16 may be involved in the action of the GOP-1. Further, the RT-PCR results showed that GOP-1 strongly up-regulate the expression of *jnk-1*, thus suggesting that the anti-aging activity of GOP-1 is possibly mediated by the *jnk-1* signaling pathway.

It is reported that HSF-1 not only cooperates with DAF-16 to activate target genes but also itself can promote longevity in *C. elegans*. We found that GOP-1 significantly up-regulated the expression of *hsf-1*, which indicted that *hsf-1* is also involved in the longevity extension effect of GOP-1. Considering the observation that GOP-1 promotes the *hsf-1* expression, it is possible that heat shock proteins (such as *hsp-16.2*) that are under the regulation of DAF-16 or HSF-1 may play a role in the stress resistance and longevity promotion of *C. elegans* treated by the GOP-1.

## 5. Conclusion

In the current study, we have shown for the first time that oligopeptide isolated from ginseng for potential anti-aging properties. Our data have clearly shown promising anti-aging activities of the GOPs, thus adding a new functional bio-activity to the ginseng. Within current study, we could identify GOPs as powerful longevity-promoting antioxidants that are worthy to be further explored for anti-aging applications in other animal systems. Further, the GOPs are interesting not only for their potent antioxidant activities to increase the nematode's resistance to fatal stress, but also for their efficacy to regulate the longevity-promoting transcription factor DAF-16 through the JNK-1 pathway. Due to the complexity and interactions of pathways involved in the regulation of aging, other mechanisms that possibly contribute to the anti-aging effects of the GOP-1 cannot be excluded.

We believe that further evaluations of the anti-aging potentials of the GOPs would be worthy.

## Conflicts of interest

The authors declare that they have no conflicts of interest concerning.

## Supplementary Material

RA-010-D0RA06093C-s001

RA-010-D0RA06093C-s002

RA-010-D0RA06093C-s003

RA-010-D0RA06093C-s004

RA-010-D0RA06093C-s005

RA-010-D0RA06093C-s006

RA-010-D0RA06093C-s007

RA-010-D0RA06093C-s008

RA-010-D0RA06093C-s009
